The article "To Explore the Diagnostic Value of Bulbocavernosus Muscle Reflex and Pudendal Somatosensory Evoked Potentials for Diabetic Neurogenic Bladder" was retracted in 2023. Reasons: unreliable results or conclusions; concerns about the data; concerns about the peer review; concerns about the citations.

# To Explore the Diagnostic Value of Bulbocavernosus Muscle Reflex and Pudendal Somatosensory Evoked Potentials for Diabetic Neurogenic Bladder

**DOI:** 10.1155/2022/6096326

**Published:** 2022-09-14

**Authors:** Ning Nan, Qi Chen, Tie Chong

**Affiliations:** Department of Urologic Surgery, Second Affiliated Hospital of Xi'an Jiaotong University, Xi'an, China

## Abstract

**Objective:**

To explore the diagnostic value of bulbocavernosus muscle reflex and pudendal somatosensory evoked potentials for diabetic neurogenic bladder.

**Methods:**

From January 2021 to December 2021, 104 patients with type 2 diabetes mellitus admitted to the hospital were recruited, with 57 allocated to the case group and 47 to the control group. Outcome measures included bulbocavernosus muscle response, pudendal somatosensory evoked potentials, and bladder residual urine volume. The connection of bulbocavernosus muscle response and pudendal somatosensory evoked potentials with bladder residual urine volume was investigated using the Pearson analysis.

**Results:**

In both males and females, the latency of the left and right bulbocavernosus muscle reflexes in the case group was longer than in the control group, but the difference was not statistically significant (*P* > 0.05), and the wave amplitude of the left and right bulbocavernosus muscle reflexes was significantly smaller than that of the control group (*P* < 0.05). The diabetic neurogenic bladder was associated with a significantly longer latency and a smaller wave amplitude of pudendal somatosensory evoked potentials versus without neurogenic bladder (*P* < 0.05). Patients with a diabetic neurogenic bladder had more residual bladder urine volume versus those without (*P* < 0.05). Bladder residual urine volume was significantly positively correlated with bulbocavernosus muscle reflex and pudendal somatosensory evoked potential latency and negatively correlated with wave amplitude (*P* < 0.05).

**Conclusion:**

The bulbocavernosus muscle reflex and pudendal somatosensory evoked potentials demonstrate great potential as adjuncts to diagnose diabetic neurogenic bladder and correlate with ultrasound results in determining bladder function in patients.

## 1. Introduction

With the aging of the population and lifestyle changes in China, the prevalence of diabetes mellitus (DM) has been increasing. Data show that there are 114 million adults with diabetes in China, the country with the largest number of diabetics [1]. By 2017, the prevalence of type 2 DM in the national survey was 11.2%, where undiagnosed diabetic patients accounted for 54% of the total number of diabetic patients. Complications of DM involve several tissues and organs such as the heart, brain, blood vessels, and kidneys and are the main cause of death and disability in its patients [2]. A common chronic complication in type 2 patients in DM is diabetic neurogenic bladder disease (DNB), in which about 50% of diabetic patients develop neuropathy, and all of these patients have a long duration of disease. The incidence of DNB in neuropathy is between 25 and 85% and is strongly related to the presence of combined diabetic peripheral neuropathy, while no correlation with the gender or age of the patient has been identified [3]. The pathogenesis is unclear, and it is considered to be caused by nerve damage or bladder dysfunction. As the disease progresses, the degree of bladder-related nerve damage will increase, resulting in lack of urinary urge and even complete absence of urination. Western medical treatment is often symptomatic, such as lowering blood glucose, nerve nutrition, and improving clinical symptoms, but fails to provide a complete cure [4, 5].

Ultrasound is currently a common clinical imaging technique. Previous research has shown that ultrasound diagnosis of bladder residual urine volume facilitates the assessment of bladder function in patients with diabetic neurogenic bladder [4] and features merits such as simplicity and a high safety profile compared to methods such as direct catheterization [5]. However, the results are easily influenced by the proficiency of the examiner [6]. Bulbocavernosus is the superficial muscle tissue that ensures the excretion of excrement from the urethra. A recent study found that bulbocavernosus muscle reflex could predict bladder voiding function [7]. Somatosensory evoked potentials are one of the objective indicators used to examine neurosensory pathway lesions. It has been reported [8] that bulbocavernosus neuropathy might primarily contribute to idiopathic overactive bladder disorder, and pudendal somatosensory evoked potentials could detect neuropathy in the external urethral sphincter and anal sphincter. The bulbocavernosus muscle reflex is caused by stimulation of the pudendal nerve, through the gingival medullary reflex arc, causing contraction of the bulbocavernosus muscle, and its latency reflects the integrity of the reflex arc composed of the peripheral afferent nerve, gingival medullary, and efferent motor fibers [9]. Therefore, abnormal reflexes of the bulbocavernosus muscle indicate potential peripheral neuropathy. Pudendal nerve somatosensory evoked potentials are generated by stimulation of the pudendal nerve generating nerve impulses that are transmitted to the cerebral cortex via the gingival medulla spinalis [10]. The potentials collected at the scalp recording electrodes showed that the length of latency and the amplitude of the somatosensory evoked potentials of the pudendal nerve are related to the function of the peripheral afferent nerves in addition to the functional integrity of the spinal cord. Thus, abnormal pudendal nerve somatosensory evoked potentials mainly reflect possible central and peripheral afferent neuropathy. Somatosensory evoked potentials of the pudendal nerves combined with the bulbocavernosus muscle reflex have localized and qualitative diagnostic significance for neurological lesions [11, 12].

However, there are few reports on bulbocavernosus muscle reflexes and pudendal somatosensory evoked potentials for diagnosing bladder function in patients with diabetic neurogenic bladder. The current study recruited 104 patients with type 2 diabetes mellitus admitted to the hospital outpatient clinic for treatment from January 2021 to December 2021, with the goal of investigating the diagnostic value of bulbocavernosus muscle reflex and pudendal somatosensory evoked potentials for diabetic neurogenic bladder.

## 2. Materials and Methods

### 2.1. Baseline Data

From January 2021 to December 2021, 104 patients with type 2 diabetes mellitus admitted to the hospital outpatient clinic for treatment were recruited, of which 57 with neurogenic bladder were assigned to the case group and 47 cases without neurogenic bladder were assigned to the control group.

The original sample size calculation estimated that 50 patients in each group would be needed to detect a 3-point difference between groups in a 2-sided significance test with a power of 0.8 and an alpha error level of 0.05.

The trial was conducted according to the Good Clinical Practice guidelines developed by the International Council for Harmonisation and in compliance with the trial protocol. The protocol was approved by the institutional review boards or independent ethics committees at each site. All patients provided written informed consent per Declaration of Helsinki principles. An independent data monitoring committee monitored safety and efficacy data. The ethics number was MI-YU20210102.

Inclusion criteria are the following: (1) aged 18 to 80 years, (2) who met the diagnostic criteria related to type 2 diabetes mellitus [9], (3) the case group met the diagnostic criteria of the neurogenic bladder [13], and (4) the case group received methylcobalamin treatment.

Exclusion criteria are the following: (1) with urinary retention or incontinence caused by drugs, prostate diseases, and other reasons; (2) with severe insufficiency of vital organs such as heart, liver, and kidney; (3) with mental, cognitive, and consciousness impairment that prevents cooperation in completing relevant examinations and treatments; (4) with the use of drugs affecting the function of the vesicourethral within the last 3 months; and (5) with neurological pathology. The baseline characteristics of the case group (25 males and 32 females, aged 39–74 years, mean age of [58.79 ± 10.32] years, duration of diabetes mellitus of [4.28 ± 2.11] years, 28 cases with oral hypoglycemic drugs and 29 cases with insulin injections in terms of diabetes mellitus medication, 21 cases with hypertension, and 18 cases with hyperlipidemia) were comparable with those of the control group (16 males and 31 females, aged 38–75 years, mean age of [59.27 ± 10.41] years, duration of diabetes mellitus of [4.32 ± 2.14] years, 21 cases with oral hypoglycemic drugs and 26 cases with insulin injections in terms of diabetes mellitus medication, 16 cases with hypertension, and 16 cases with hyperlipidemia) (*P* > 0.05).

### 2.2. Treatment

#### 2.2.1. Bulbocavernosus Muscle Reflex [14] Measurement

With the patient in a lithotomy position, the saddle stimulation electrode was connected to the pubic symphysis, the grounding electrode was placed on the thigh, and the recording electrode was a concentric needle inserted into the bulbocavernosus muscle on the left and right sides of the patient. The full-function EMG evoked potentiometer (Dandy, Denmark, KEYPOINT) was activated using square wave stimulation with a frequency of 1.9 Hz, stimulation intensity was set to 7 times the sensory threshold, and 20 reflected waves were recorded. The scanning time was 5 ms/div, the analysis time was 100 ms, the bandwidth was 10–2000 Hz, and the latency and wave amplitude were calculated.

#### 2.2.2. Pudendal Somatosensory Evoked Potentials [15] Measurement

The position of the patient and the placement of the stimulating electrode were the same as 1.2.1. The recording electrodes were concentric needles, placed in the Cz-2 area of the scalp to record scalp potentials, and the reference electrode was placed in the Fz area. The full-function EMG evoked potentiometer was activated using the square wave stimulation, with electrode impedance <5 k*Ω*, stimulation intensity set to 3 times the sensory threshold, and analysis time of 100 ms, and P41 wave latency and wave amplitude were calculated.

#### 2.2.3. Measurement of Residual Bladder Urine Volume by Ultrasound

After drinking 300 mL of water before the examination, an ultrasound was performed after forceful urination, and the maximum anterior and posterior diameters, upper and lower diameters, and left and right diameters of the fluid dark area in the bladder were measured. The residual bladder urine volume (mL) = anterior and posterior diameters × upper and lower diameters × left and right diameters × 0.52.

### 2.3. Statistical Analysis

The mean difference between the two groups was tested using the Student's *t*-test for normally distributed variables and Mann-Whitney *U* test for nonnormal variables.

SPSS 20.0 software was used for data analyses. Normally distributed measurement data were expressed as ($\bar{x}\pm s$) and subject to independent samples *t*-test. Count data were expressed as frequencies or composition ratios and were examined by chi-square test. Correlations were analyzed using the Pearson analysis. A difference was considered statistically significant at *P* < 0.05.

## 3. Results

### 3.1. Bulbocavernosus Muscle Reflex

In both males and females, the latency of the left and right bulbocavernosus muscle reflexes in the case group was longer than in the control group, but the difference was not statistically significant (*P* > 0.05), and the wave amplitude of the left and right bulbocavernosus muscle reflexes was significantly smaller than that of the control group (*P* < 0.05) (Table 1).

### 3.2. Pudendal Somatosensory Evoked Potentials

The diabetic neurogenic bladder was related with a substantially longer latency and a lower wave amplitude of pudendal somatosensory evoked potentials in both males and females compared to those without neurogenic bladder (*P* < 0.05) (Table 2).

### 3.3. Bladder Residual Urine Volume

Patients with a diabetic neurogenic bladder exhibited greater residual bladder urine volume in both males and females than those without a diabetic neurogenic bladder (*P* < 0.05) (Table 3).

### 3.4. Correlation Analysis

The volume of remaining pee in the bladder was substantially linked with the bulbocavernosus muscle response and the latency of pudendal somatosensory evoked potentials, but not with wave amplitude (*P* < 0.05) (Table 4).

## 4. Discussion

Neurogenic bladder refers to significant damage to the nerves that govern the normal physiological function of the bladder, resulting in lower urinary tract disorders and complications [16]. The core symptoms of the disease are changes in urine volume and frequency and dyspareunia, accompanied by many clinical manifestations such as urinary retention and urinary tract infections, which are prone to cause damage to the renal function of the patient without professional care treatment and may pose great threats to the life safety of the patients [17]. With lifestyle changes, the underlying elements of stroke, diabetes, and spinal cord injury are on the rise, leading to a rapid increase in the ultimate scale of the disease. In clinical practice, neurogenic bladder reduces patients' personal quality of life scores to varying degrees and also poses an obstacle to the diagnosis and treatment of various primary conditions as well as to the rehabilitation of patients [18, 19]. The early symptoms of the neurogenic bladder are insidious, mostly including mild symptoms of urinary difficulty, frequency, and urgency [20], resulting in delayed diagnosis and a poor prognosis in most cases [21]. Research has demonstrated that voiding symptoms and urinary urgency were associated with high post-void residual urine volume in men and slow urine flow and terminal dribbling are associated with residual urine volume in women [22]. The morphological features in the bladder cavity may be readily seen with ultrasound, and the bladder residual urine volume can be determined by measuring the right and left, upper and lower, and anterior and posterior bladder diameters after urination [23]. However, ultrasound results are susceptible to subjective factors and are associated with a certain missed diagnosis rate [24]. Therefore, there exists an urgent need to explore new examination methods for the diagnosis and prognosis of diabetic neurogenic bladder.

Bulbocavernosus muscle reflex is a test that is performed by stimulating the male penile and female clitoral nerves, via the sacral medullary reflex arc, which consequently causes bulbocavernosus muscle contraction and is mainly used to diagnose peripheral neuropathy [25]. Pudendal somatosensory evoked potentials are an examination to assess pelvic floor function by recording scalp Cz-2 area potentials and calculating P41 wave latency and wave amplitude [26]. Given the sex differences, the patients in the two groups were further subgrouped by sex, and the results of the present study showed that in both males and females, the latency of the left and right bulbocavernosus muscle reflexes in the case group was longer than in the control group, but the difference was not statistically significant, and the wave amplitude of the left and right bulbocavernosus muscle reflexes was significantly smaller than that of the control group, which may be attributable to the predominance of axonal damage in the pubic neuropathy in patients with diabetic neurogenic bladder, which is consistent with the results of previous research [27], and patients with neurogenic bladder showed more severe pubic neuropathy and vesicourethral dysfunction compared to those without neurogenic bladder. The bulbocavernosus reflex is caused by stimulation of the dorsal nerve of the penis and the efferent nerve via the sacral medullary S2 to S4 reflex arc, causing contraction of the bulbocavernosus and sciatic cavernosus muscles. Parasympathetic excitation causes relaxation of the cavernous smooth muscles and cavernous arteries of the penis, the parasympathetic nerves can be transmitted to the cavernous nerves through the visceral nerves of the lower abdominal pelvis and the pelvic plexus, and somatic nerve stimulation acts on the pubic motor neurons to produce contraction of the bulbocavernosus and sciatic cavernosus muscles [28].

Moreover, in both males and females, the diabetic neurogenic bladder was associated with a significantly longer latency and a smaller wave amplitude of pudendal somatosensory evoked potentials versus without neurogenic bladder, indicating a possible association between the occurrence of diabetic neurogenic bladder and peripheral neuropathy. Ultrasound measurement of bladder residual urine volume revealed that in both males and females, patients with a diabetic neurogenic bladder had more residual bladder urine volume versus those without a diabetic neurogenic bladder, which was associated with urinary retention due to perivaginal neuropathy and was consistent with previous findings [29]. Diabetes, chronic alcohol consumption, and vitamin deficiencies frequently cause peripheral nerve axon spontaneity and/or demyelination, affecting the synthesis and release of neurotransmitters. However, with the exception of men with spinal cord injury, the amount of data on treatment options for different neurological disorders remains scarce. Despite abnormalities of the bulbocavernosus muscle reflex as an important factor in neurogenic bladder, treatment efficiency remains unsatisfactory. Furthermore, bladder residual urine volume was significantly positively correlated with bulbocavernosus muscle reflex and pudendal somatosensory evoked potential latency and negatively correlated with wave amplitude, suggesting that bulbocavernosus muscle reflexes and pudendal somatosensory evoked potentials correlate with ultrasound in determining bladder function in diabetic patients and may be an aid in diagnosing diabetic neurogenic bladder, thus improving the early diagnosis rate.

This study has the following shortcomings: 1. The sample covered 18–80 years old, which failed to achieve reliable observation for the whole patient population. 2. The sample size of this study is relatively small, resulting in a certain risk of error, and future studies with an increased sample size are required to improve the feasibility of the analysis results. 3. The follow-up was short, and no long-term efficacy data was available.

In conclusion, the bulbocavernosus muscle reflex and pudendal somatosensory evoked potentials demonstrate great potential as adjuncts to diagnose diabetic neurogenic bladder and correlate with ultrasound results in determining bladder function in patients.

## Figures and Tables

**Table 1:** Comparison of bulbocavernosus muscle reflex ($\bar{x}\pm s$).

Groups	*n*	Latency (ms)		Wave amplitude (mV)	
		Left	Right	Left	Right
Case group					
Male	25	55.37 ± 14.36	56.43 ± 13.66	0.18 ± 0.05^a^	0.23 ± 0.03^a^
Female	32	55.46 ± 14.41	57.11 ± 13.69	0.21 ± 0.04^a^	0.19 ± 0.05^a^

Control group					
Male	16	53.68 ± 14.52	55.98 ± 13.63	0.49 ± 0.11	0.54 ± 0.13
Female	31	54.21 ± 14.47	56.39 ± 13.58	0.51 ± 0.06	0.49 ± 0.15

Note: a suggests a significant difference (*P* < 0.05) in comparison with same-sex controls.

**Table 2:** Comparison of pudendal somatosensory evoked potentials ($\bar{x}\pm s$).

Groups	*n*	Latency (ms)	Wave amplitude (mV)
Case group			
Male	25	44.52 ± 3.11^a^	1.28 ± 0.84^a^
Female	32	43.38 ± 2.97^a^	1.33 ± 0.86^a^

Control group			
Male	16	41.23 ± 3.14	1.54 ± 0.86
Female	31	40.57 ± 2.88	1.58 ± 0.85

Note: a suggests a significant difference (*P* < 0.05) in comparison with same-sex controls.

**Table 3:** Comparison of bladder residual urine volume (mL, $\bar{x}\pm s$).

Groups	*n*	Bladder residual urine volume
Case group		
Male	25	189.85 ± 44.87^a^
Female	32	192.98 ± 46.46^a^

Control group		
Male	16	54.23 ± 21.76
Female	31	51.98 ± 22.34

Note: a suggests a significant difference (*P* < 0.05) in comparison with same-sex controls.

**Table 4:** Correlation of bulbocavernosus muscle reflex and pudendal somatosensory evoked potentials with bladder residual urine volume.

Examinations	Indices	*r*	*P*-value
Bulbocavernosus muscle reflex	Latency	0.128	0.024
	Wave amplitude	−0.113	0.036
Pudendal somatosensory evoked potential	Latency	0.236	0.008
	Wave amplitude	−0.192	0.011

## Data Availability

All data generated or analyzed during this study are included in this published article.
